# The Chain Mediating Effect of Network Behavior and Decision Self-Efficacy between Work Skills and Perceived Employability Based on Social Cognitive Theory

**DOI:** 10.1155/2022/5240947

**Published:** 2022-10-04

**Authors:** Liping Yang, Hong Zhang

**Affiliations:** ^1^International College, National Institute of Development Administration, Bangkok 10240, Thailand; ^2^Institute of Social Technology, Suranaree University of Technology, Nakhon Ratchasima 30000, Thailand

## Abstract

The purpose of this study is to investigate the chain mediating effects of networking behaviors and decision self-efficacy between work skills development and perceived employability. Structural equations modeling is used to analyze data collected from 813 Chinese students. The results show the following: first, the work skills development is positively correlated with perceived employability. Second, network behavior and decision self-efficacy each have a mediating effect between work skills development and perceived employability. Finally, this study found a chain mediating effect of network behavior and decision self-efficacy between work skills development and perceived employability. Therefore, this research shows that Work-Integrated Learning (WIL) needs to focus not only on skills development and employability outcomes but also on developing a strong network-based platform for stakeholders. In addition, higher education institutions and workplaces should also provide career guidance and counseling centers to help students build confidence in career decision-making and ensure students' mental health care and healthy career development.

## 1. Introduction

Work skills are essential to people's mental health care. A survey revealed nine work skills in the Indian healthcare industry. They found that with changing supply and demand patterns and customer demand for service excellence, workplaces are increasingly seeking greater proficiency, a serious challenge in today's era. Hence, organizations expect employees to have excellent employability skills. They also found that, in the healthcare industry, employee work skills were positively correlated with patient satisfaction. Therefore, the healthcare industry also needs to train effective work skills to remain competitive [1]. Network behavior described a form of network-based social support, and it has always been closely associated with students' mental health issues. One study used four scales, the Symptom Checklist 90 (SCL-90), the Teacher–Student Relationship Questionnaire (TSRQ), and the Peer Relationship Scale (PRS), and assessed psychological symptoms, quality of teacher–student relationships, and quality of peer relationships. They found that risk from all types of psychological symptoms was associated with school ties. Furthermore, poor school relationships carry a high risk of mental health problems. So they suggested that school administrators should urgently improve students' school relations [2]. In fact, communication skills in work skills are positively related to self-efficacy. In addition, superior communication skills can aid in treatment and effective care in the healthcare industry, and training courses in communication skills help improve self-efficacy [3]. And then, career decision-making self-efficacy helps to improve the emotional life quality of students. Higher career decision self-efficacy leads to more positive emotions [4]. Furthermore, perceived employability is a crucial psychological protection resource. It reduces the psychological distress and worry of work seekers due to employment difficulties and also reduces the current fears caused by COVID-19 and it promotes market prosperity. Therefore, colleges and universities should improve the employability of students. For example, career guidance and training to improve students' employability [5]. This study analyzed the relationship between work skills and perceived employability from the perspective of mental health care. Work skills development cultivates the employability of university students, and good employability is an important driving force for students' future career success. Currently, perceived employability places new demands on work skills development. However, most of the current research and discussions in this area focus on the assessment of work skills development [6], students' skills for coping with work readiness [7], the application of work skills development models [8], curriculum mapping [9], and whether work skills development can affect graduate employability [10, 11]. We need to focus on skills development. Because the past study has shown that the ownership of employability skills has the possibility to find out satisfactory careers for students, because they will be even more employable in their working livelihood [12]. Therefore, healthy career success benefits students' mental health care.

Based on social cognitive theory, the implementation of skills must be varied to fit changing environments and serve multiple aims. Cognitive training affects the beginning and middle stages of skill development. The structure of knowledge determines how to select the right skills to achieve specified goals. Continued training makes the skills easy to apply, leading to a certain level of competence [13]. Work skills development can be used as a tool for viewing student progress, and students can use it to assess their own skill levels [6]. Whereas perceived employability involves the person's feeling of his or her probabilities of gaining and keeping employment [14]. Employers value the soft skills of graduates more, and universities can be more inclined to develop soft skills courses, which can improve their employability. As a result, graduates can demonstrate soft skills to employers when they are looking for a job [10]. Consequently, it is in the best benefit of students to acquire new skills and knowledge as this is significant for their employability [15]. This study revealed a new framework for the relationship between work skills development and perceived employability that incorporates network behavior and decision self-efficacy as mediators and uses quantitative methods to verify chain mediation effects, complementing knowledge about the relationship between these variables. Furthermore, the present study has described new knowledge of these cognitive developmental processes and found that work skills development improves perceived employability by enhancing network behaviors to shape confidence in decision self-efficacy. In summary, past research has emphasized the impact of work skills on employability but has not incorporated both network behavior and decision self-efficacy into the research framework. Furthermore, this study first validates the reliability and validity of the network behavior scale and decision self-efficacy scale in a Thai environment, providing a measurement tool for future researchers.

## 2. Literature Review

Social cognitive theory (SCT) argued that the agents who strive to improve the quality of life and the environment are individuals [16]. Individuals are apt to seek their targets if they think their own capabilities and actions are able of meeting the wished outcomes [17]. Work skills development helps increase their cognition, continuously strengthen their skills and knowledge, and make their network behavior more exploratory, systematic, and meaningful for career development. This research used the SCT to inspect how students in work skills development can improve their capability to decision self-efficacy through network behavior, which in turn influences students' perceived employability. Employability often helps employees be flexible to changes in the work environment to societal and human resource and is explained as features that develop adaptive thinking, actions, and affections that aid personals counter flexibly to alterations in their task circumstance [18]. Therefore, persons with strong employability have a propensity to be buffered against passive influences of unemployment [18, 19]. Furthermore, some respects of employability assist persons with winning work recovery. First, one of the secrets to people's ability to stay employed is to have strong work skills and ongoing training, which enables them to find new jobs [18]. Next, people with sufficient social capital can access more resources in professional networks [20]. Social capital offers job hunters precious chances; social connections can cause job hunters to notice vacancies, bringing to “accidental job chance” [21]. Because knowledge derived from social relationships is positively correlated with people's job fit. When people meet talented insiders, they will gain a more precise view of future work [22]. Therefore, the number of informal career networks remains positively correlated with potential job opportunities and helps people gain greater employment competitiveness [23].

Social cognitive theory (SCT) describes the social transmission of new behavioral patterns [24]. It mainly includes the acquisition of knowledge, the innovation and practice of thinking, and the functional value of these elements. Its function also concerns utilization determinants. In fact, many factors, containing perceived self-efficacy to have a good command of the necessary abilities, ownership of basic resources, and outcome expectations, are related to the benefits and costs of new behavioral patterns, and the key factor that people practice is their perceived barriers and potential opportunities. In addition, social networking is also a major feature [25, 26]. Structural interconnectedness offers latent routes of affect; psychosocial factors greatly decide the destiny of what diffuses by those gregarious networks [13]. Perceived self-efficacy can directly or indirectly influence behavior, so it is critical in SCT [27, 28]. In addition, self-efficacy also positively affects people's motivation for outcome expectations [29–31]. In fact, self-efficacy determines how choices and decisions are made. For example, when people make decisions that do not ensure the success of the predetermined plan and are firmly maintained, especially when people encounter difficulties, it is important for individuals to make decisions with self-confidence [32]. Therefore, confidence based on support and maintenance efficacy is the key to action psychology, and decision psychology needs its support [33].

According to attribution theory, human motivation can be influenced by the attribution of their performance [34]. Because people often assess whether their expectations are being met, and use the results of those assessments to guide their actions. When people imagine themselves in a situation of success, it means that they have strong efficacy, so the guidance of this efficacy positively promotes their performance and behavior. Conversely, self-doubting people impair their performance because they lack self-efficacy. In addition, when people are doing evaluations, high-performing people are more proactive in pursuing opportunity value [35, 36]. On the other hand, highly productive people have strong strategic sensitivity and high cognitive abilities that help them monitor their living environment more effectively [37]. In addition, people with high self-efficacy are better at asking deep and broad questions, and as a result, they are able to save more time, which is an easy strategy for acquiring knowledge [38].

This study also investigates whether network behavior affects decision self-efficacy. Regarding network behavior, it usually means that a person has a social relationship or a willingness to connect with others. According to social cognitive theory (SCT), SCT emphasizes the concept of collective agency. A central part of the collective agency is that people have confidence in collective strength and the ability to achieve desired outcomes. In other words, collective performance is the result of everyone's efforts [13]. In conclusion, collective self-confidence is positively correlated with people's achievement [39]. High self-efficacy always helps to coordinate and improve collective performance, both at the social and individual levels [13].

### 2.1. The Influence of Work Skills Development on Perceived Employability

The impact of work skills on employability is very significant because work skills bring competitiveness. For skills development, Chandran [40] described many recommendations like devising a new course, making new teaching outlines, running English word coaching plans, mixing general skills and technological skills, and conforming soft skills into the course to give the power to students with employability. In fact, graduates demand to be competitive to guarantee they can survive in the labor market. To be competitive, well-educated graduates demand to hold themselves with skills. These skills can be a feature to them, and they can decide their marketability [41]. According to Jackson [42], WIL is a tool that enhances graduate work practice and has been shown to improve graduate work skills and employability. Work skills include a range of skills that are used on the job, studies have pointed out that language skills have a positive impact on the employability of international graduates in Norway, and graduate employability is influenced by many work skills such as social skills, communication skills, IQ, and network skills, etc. These work skills all affect the employability of graduates [43]. When it comes to employability, what matters most is the link between a job seeker's skills and an employer's needs [44]. Business skills in work skills greatly influence employability, especially for business students. Different employers need different job skills. Some employers are very obsessed with the IT skills of job seekers, some employers pursue business-related skills, and some employers need soft skills on the job, such as coordination and communication skills. Some employers require graduates to have office skills such as writing and communication skills, creative and critical thinking skills, and more. Most employers also attach great importance to the actual work experience of graduates, and graduates who have work experience or participated in job placement programs are more concerned employers. In addition, political skills have positive implications for student's entrepreneurial education [45]. Therefore, for work skills development, both hard skills and soft skills are core aspects that reflect the employability of graduates [46]. Therefore, we propose Hypothesis 1.

**Hypothesis 1 .**

There will be a positive relationship between work skills development and perceived employability.

### 2.2. Mediating Role of Networking Behaviors

Batistic and Tymon [47] demonstrated that networks arise from frequent access to resources and information, and it contributes to increased perceived employability. Chen [48] proposed that social networks help graduates improve their employability. University graduates ought to attach importance to the forming of studying conduct based on a sociable network to enhance their employability in China. Craig [49] confirmed that robust ways for improving employability ought to be executed to create even more skilled or equipped employees, such as offering chances for an internship, networking, and short curriculums. In addition to the industry and internship interchange, networking and response for the student are same significant for student's employability [40]. The principle of network behavior is like the knowledge creation process. The knowledge creation process is to share individual ideas, transform scattered tacit knowledge into explicit knowledge shared by organizations, and finally store knowledge in a database to integrate this scattered knowledge [50]. Network behavior is a key career strategy because it means that people have the potential to communicate and connect with potential employers ahead of time for potential employment opportunities. In addition, career outcomes were also associated with online behavior [51]. Networking is explained as a target-guided activity which happens both internally and externally in a team, concentrated on building, developing, and using relationships. Moreover, that is affected by various kinds of person, work, and team level reasons and bring about to advanced reputation and authority, work outcomes, teams gain strategic intelligence and professional success. Therefore, it is held to be of a large career worth for aspirants or organized system [52]. In fact, the moderation of skill development and network behavior was positively associated with perceived employability [53]. Some studies have tested the influence of the superior–subordinate relationship on employees' emotions, and the research shows that the manager's work autonomy has a positive moderating effect on the relationship [54]. Therefore, maintaining a good interpersonal network has a positive significance for people's lives, and network behavior is conducive to people's good performance. Therefore, we propose Hypothesis 2.

**Hypothesis 2 .**

Network behavior plays a mediating role in the associations between work skills development and perceived employability.

### 2.3. Mediating Role of Decision Self-Efficacy

Makki et al. [55] found that engineering graduates had higher skill levels, had high self-efficacy, and were more eager to explore their career plans. In addition, universities can develop relevant training for them, making them highly employable. Therefore, getting enough work preparedness skills, and cultivate graduates' confidence in their abilities, will guide them toward valid exploration of career selections [56]. Perceived employability (PE) is people's viewpoint of their easy access to employment, and it is positively related to self-efficacy (SE) [57]. PE and SE are distinct but related [58]. Employability is a significant reason that can decide the quality of future graduates, Tentama and Nur [59] explored the role of SE and partner interaction on student employability. They reported SE is positively related to PE [60]. Moreover, Sultana and Malik [61] found that self-efficacy also promotes protean person to develop high perceived internal and external employability. They described the expectation of full mediation of SE on PE. Charoensukmongkol and Pandey [62] pointed that the mediating effect of sales self-efficacy between cultural intelligence and the quality of cross-cultural sales presentations. These positive effects also reflect the objectivity of self-efficacy in improving people's work quality and performance. Therefore, we propose Hypothesis 3.

**Hypothesis 3 .**

Decision self-efficacy (DSE) has a mediating role in the associations between work skills development (WSD) and perceived employability (PE).

### 2.4. The Chain Mediating Effect of Network Behavior and Decision Self-Efficacy

The present study has discussed the relationship between DSE and career exploration. Brown et al. [63] stated that career decision self-efficacy can lead to sustainable careers. Chen et al. [64] concluded that DSE positively predicts sustainable career development. Therefore, self-efficacy and work experience play a key role in students' career development [65]. Career decision self-efficacy predicts the purpose of career exploration [66]. Lack of participation affected career exploration and, furthermore, career self-efficacy had an impact on self-exploration [67]. People need to improve DSE for more work outcomes and sustainable career development [68]. Parents and teachers can actively contribute to DSE [69]. Program participation was positively correlated with DSE, and in addition, career help and support from school staff, as well as career-related connections and activities, supported participants' DSE [70]. In addition, nontraditional university women with children were more likely to network with shared interests, and these network behaviors were also associated with higher levels of DSE [71]. Lastly, those who felt responsible for others' happiness also highly showed levels of DSE [72]. Therefore, with more beneficial interpersonal relationships they can brook more unpredictability and uncertainty when they make decisions. Evidently, great social bonds and great social functioning can promote their capability of controlling the future [73]. For instance, Pond and Hay [74] reported that the provision of information enhanced self-efficacy. Similarly, it could use by government employees doing organizational restructuring [75]. Network diversity can be in various contexts, such as family and friends, partnerships, someone's advice, and the same purpose of interest [76]. Degree centrality quantifies the relative number of individuals in a team, and it represents how closely an individual is connected to other people in the network [77]. Therefore, degree centrality is positively related to the number of relations in the network. Based on SCT, degree centrality confers information richness and social support [78]. Instead, this should provide a better level of confidence during the transition. The centrality of social networks establishes self-efficacy [79]. Therefore, we propose Hypothesis 4.

**Hypothesis 4 .**

Network behavior and decision self-efficacy will have a chain mediating effect between work skill development and perceived employability. In conclusion, this study has four hypotheses, as shown in Figure 1.

## 3. Research Methods

### 3.1. Respondents

Our respondents were from the Yunnan University of Business Management in Yunnan Province, China. The location was chosen because Yunnan Province has carried out higher education school-enterprise cooperation “going out” activities [80], so this study could test university students' learning outcomes and have a practical significance in the results. Second, given the good communication between us and the university, the university agreed to participate in the sampling of this study, so there is convenience and transparency in the study. Questionnaires were distributed to 1252 Chinese undergraduate students, and 813 valid questionnaires were returned, with a recovery rate of 65%. Among the interviewees, men accounted for 25.6%, women accounted for 74.4%, and there were more women than men. Young people aged 16 to 19 accounted for 44% and aged 20 to 23 accounted for 56%. Respondents are undergraduate students in various majors; 100% are undergraduates and below, 4.5% are Economics and Business students, followed by Engineering 5.9%, Humanities and Arts 61.4%, and Science 28.2%.

### 3.2. Procedure

The subjects of this study are Chinese undergraduate students. Respondents participated in work or internship programs to varying degrees. Participants receive support from employers and schools in terms of internships in the workplace, work skills, and other needs. The issues involved in this study have been well understood by the respondents and can meet the criteria of empirical analysis. In April 2021, we communicated with the staff members in charge of the Work-Integrated Learning (WIL) internship program at the university and sent an invitation to participate in this research to their students via e-mail. We inform students that these data will be used for research purposes only and that students' personal privacy is kept confidential. In addition, students have the right to choose whether to participate in this research, and they can stop or refuse to participate at any time during the research process. We only provide access to the return form for students who would like to participate in research.

### 3.3. Measures

To ensure the reliability and validity of the study, the study referred to important relevant literature and selected four authoritative scales. This study summarizes the previous literature, combined with the specific scenarios of WIL, and uses the work skills development scale and the networking behaviors for career development scale, the decision self-efficacy for career exploration scale, and the perceived employability scale, so that the measurement is suitable for students and finally forms a scale. A five-point Likert scale was used in the present study, and undergraduate students evaluate the corresponding items according to their actual conditions.

#### 3.3.1. Work Skills Development

The work skills development measured in this study is mainly based on the students' personal level. We asked students to rate themselves on a 5-point Likert scale. The lowest value is 1 = not developed, 5 = very well developed. The 21 items are: Communication Skills; Writing Skills; Professionalism in Your Field; Interpersonal Skills; Leadership Skills; Teamwork and Cooperation; Analytical Skills; Initiative; Decision Making Skills; Problem Solving Skills; Flexibility; Self Confidence; Self-Control; Ability To Work Independently; Time Management; Ability and Willingness to Learn; Achievement Orientation; Resilience Skills; Conflict Management; Prioritization, quality, and accuracy of the work; Networking and collaborating in virtual environments [81]. The results of the study showed that the scale's Cronbach's alpha coefficient was 0.968, so it had very high reliability.

#### 3.3.2. Networking Behavior

The scale was used to assess students' career development network behavior. This scale include “I use computers and connections for easy access to employment opportunities; I use many networking tools such as WeChat, Twitter, line, etc. to build connections or get in touch with celebrities in other industries, which facilitates my professional network; Mentors are great and they provide great advice on careers; I have great relationships with people from government agencies who offer good career advice and give me employment opportunities; I talk to family and friends about careers activities to promote the search for more employment opportunities; I am good at using computer networks to contact people of the same major as me; I am good at using social networking tools to promote the realization of my ideal career;I'm good at using the Internet and learning from it; I'm good at using the Internet to advance career skills; I am good at using the Internet to find a job.”10 items. These items are translated into English sentences that are more suitable for Chinese people to understand. The results of the study showed that the scale's Cronbach's alpha coefficient was 0.930, so it had high reliability.

#### 3.3.3. Decision Self-Efficacy

This scale was made by Lent et al. [82]. The scale is measured by 12 items, A 5-point rating scale will be used to rate each item (1 = no have confidence, 5 = highest confidence). The results of the study showed that the scale's Cronbach's alpha coefficient was 0.942, so it had high reliability.

#### 3.3.4. Perceived Employability

This scale measures perceived internal employability by Rothwell et al. [83]. Räty et al. [84] used this scale to measure the employability and self-perception of Finnish university students. The scale has been validated in countries such as Turkey [85], Spain [86] and Finland [87]. The developed scale includes seven items. For example: “The labor market has generally a high demand for graduates at the moment,” “There are plenty of job vacancies in the geographical area in which I am looking,” “I can easily find out about opportunities in my chosen field,” “The skills and abilities I possess are what employers are looking for.” These seven items measure the students' Self-perceived employability. The results of the study showed that the scale's Cronbach's alpha coefficient was 0.887, so it had high reliability.

#### 3.3.5. Control Variables

Since both age and gender variables are not related to the hypothesized variables, so the study excluded the effect of control variables.

## 4. Results Analysis

This research uses data analysis tools such as SPSS v23 and Mplus v8.3. The research is mainly analyzed in three stages: first, the model fit, reliability, and validity of the measurement model are analyzed; second, descriptive statistics are used for the research variables; and finally, we tested the chain mediation effect based on the structural equation model of Mplus v8.3 (Model 6) created by Hayes [88].

### 4.1. Common Method Deviation

Based on Harman's univariate method to test, using the confirmatory factor analysis (CFA), so we ran all measures fixed on one underlying factor and the results showed poor fit (*χ*^2^ = 10586.684, *df* = 1175, *χ*^2^/*df* = 9.010, CFI = 0.695, TLI = 0.682, RMSEA = 0.099, SRMR = 0.087) [89], the results indicated that most of the variation could not be explained by methodological factors [90]. In addition, this study also used exploratory factor analysis (EFA) that is performed without rotation. The results show that the cumulative explained total variance is 45.930%. The first factor explained less than 50% of the variance [91]. Therefore, this study did not find serious common method bias.

### 4.2. Confirmatory Factor Analysis

We performed a CFA for each variable by Mplus v8.3 to analyze the discriminant validity of all variables. As shown in Table 1, the fit of the four-factor model assumed is the most ideal and all meet the standard, while the fit of other factor models is relatively poor.

### 4.3. Descriptive Statistics and Correlation

Statistical analysis of the mean, standard deviation, and correlation coefficient of the latent variables was performed using SPSS v23. As shown in Table 2, the study found significant correlations between work skills development, network behavior, decision self-efficacy, and perceived employability.

### 4.4. Convergent Validity and Discriminant Validity Test

The AVE values corresponding to the four factors are greater than 0.5, and the CR values are higher than 0.7, which means that the data have good convergent validity [92]. As shown in Table 3, using the HTMT value for discriminant validity analysis, all HTMT values are less than 0.85, which means that the factors have good discriminant validity [93]. The study used SPSS v23 for exploratory factor analysis, fixed the number of four factors, and set the maximum variance rotation method (Varimax) to rotate the data. The KMO value is 0.977 > 0.9 (*p* < 0.001), Bartlett's Test of Sphericity passed, and the measurement relationship of the factors is good, as shown in Table 4. These results explain the relationship between the variables and provide more evidence for more analyses.

### 4.5. Structural Equation Modeling Analysis

First, construct a structural equation model 1, and the main effect is tested, with work skills development as the independent variable and perceived employability as the dependent variable. The fitting index of model 1 meets the requirements (*χ*^2^*/df* = 4.912, CFI = 0.919, TLI = 0.912, AIC = 40310.175, BIC = 40709.737, SRMR = 0.0354, and RMSEA = 0.069); therefore, the model is fitted. The main effect test results show that work skills development has a positive effect on perceived employability (*β* = 0.526, *p* < 0.001), and supports H1. Second, the establishment of Model 2 and Model 3 regards the network behavior and decision self-efficacy as single mediators. The results show that the model is fitted (model 2: *χ*^2^*/df* = 4.066, CFI = 0.912, TLI = 0.906, AIC = 2849.672, BIC = 3221.029, SRMR = 0.0353; RMSEA = 0.061; model 3: *χ*^2^*/df* = 3.982, CFI = 0.910, TLI = 0.905, AIC = 3100.992, BIC = 3491.153, SRMR = 0.0340; RMSEA = 0.061). Through Mplus v8.3, the bootstrap method is used to repeatedly sample 5000 times to test the mediation effect. For model 2, the mediating effect of network behavior was 0.361, with a 95% confidence interval [0.303, 0.429], excluding 0, based on the assumption that H2 was verified. For model 3, the mediating effect of decision self-efficacy is 0.384, with a 95% confidence interval [0.320, 0.455], excluding 0, based on the assumption that H3 is verified.

Finally, the chain mediation effect was tested. A correlation was observed between the two mediator variables in network behavior and decision self-efficacy. The study hypothesized that these two variables have a chain mediating effect between work skills development and perceived employability. According to Mplus v8.3, the 95% confidence interval of the mediating effect was estimated by extracting 5,000 bootstrap samples, and the chain mediation effect of network behavior and decision self-efficacy was tested significantly, as shown in Figure 2. Work skills development ⟶ network behavior ⟶ perceived employability mediating effect is 0.241, 95% confidence interval is [0.194, 0.297], excluding 0, and mediating effect is significant. Work skills development ⟶ decision self-efficacy ⟶ perceived employability, the mediating effect is 0.142, the 95% confidence interval is [0.106, 0.184], excluding 0, and the mediating effect is significant. Work skills development ⟶ network behavior ⟶ decision self-efficacy ⟶ perceived employability, the chain mediating effect is 0.120, 95% confidence interval [0.092, 0.156], excluding 0, indicating that networking behavior and decision self-efficacy are between work skills development and perceived employability, and H4 is verified. The results are shown in Table 5.

## 5. Conclusions

### 5.1. Research Conclusions

This research explores the influence mechanism of work skills development on perceived employability based on social cognition theory. The structural equation modeling (SEM) is used to test the individual and continuous mediation effects of networking behavior and decision self-efficacy at the same time, and to verify the ability of students' networking behavior and decision self-efficacy. The multi-chain-based mediation role in the perceived employability relationship provides a new path mechanism for considering the influence of work skills development on perceived employability. Empirical research shows the following results: (1) Main effect test. The results show that there is a positive correlation between work skills development and perceived employability. (2) Mediating effect test. The test results show that networking behavior and decision self-efficacy play a mediating role in work skills development and perceived employability, respectively. Networking behavior enhances the ability of decision self-efficacy for career exploration and plays a continuous mediating role in the impact of work skills development on perceived employability.

### 5.2. Theoretical Implications

These findings allow us to understand how work skills acquired in Work-Integrated Learning (WIL) correlate with perceived employability and answer the question of whether network behavior, decision self-efficacy, and employability are perceived. Work skills development not only provides social capital such as soft skills but can also improve students' attitudes towards interpersonal networks and confidence in decision-making, thereby enhancing their perception and self-evaluation of employability. First, work skills development and skills that employers perceive as critical to the workplace help reduce the gap in producing high-skilled graduates [94]. And then, students try to connect with others who have the ability to provide work or work assistance [51], for example: through networking (i.e., friendships, parental support, teacher connections) [69], project participation, the ecosystem of career-related activities and other interpersonal activities enhance their decision self-efficacy [70], and the higher the self-efficacy, the naturally improved perceived employability [60]. Therefore, with good interpersonal relationships, students can make decisions more calmly. Clearly, good social bonds can enhance their abilities [73].

We take a unique approach to understand how work skills development affects perceived employability. Structural equation modeling was used to examine the multiple mediating roles of network behaviors and decision self-efficacy (DSE) between work skills development and perceived employability, elucidating the impact of career network behavior and DSE on work skills development, and clarifying the specific path and internal mechanism of career network behavior and DSE in the impact of work skills development on perceive employability. The research results verify that work skills development shapes confidence in DSE by reinforcing network behaviors and that during these cognitive developmental processes, major factors that enhance perceived employability are revealed.

### 5.3. Managerial Implications

Work-Integrated Learning (WIL) could improve students' employability skills, including real work skills [95], and soft skills [96, 97]. Students, as the main stakeholders of WIL, should consider their own career planning, and students should focus on work skills development, including the training of hard and soft skills for themselves. In addition, students can actively build their own various interpersonal networks during the process of internship [76]. When they are confused about their careers, they could seek career help and support from friends, family members, colleagues, schools, mentors, employers, etc., and build relationships in advance for their career decisions. At the same time, these network connections also help students' judgment ability for career exploration, so students can gain sufficient decision-making confidence and enhance their decision self-efficacy [69]. Students could focus on their work skills and could rely on strong social network relationships and decision self-efficacy to enhance their perception of employability. Therefore, these students could achieve career success in the future. In addition, this study suggested that when conducting WIL, colleges and universities should not only focus on work skills and employability but also actively help students develop interpersonal network relationships, such as the establishment of teacher–student relationships, workplace boss–student relationships, colleague–student relationships, and academic tutor-student relationship. At the same time, colleges and universities should provide more career guidance and advice for students participating in WIL. Taken together, these learning outcomes benefit student mental health care and career development.

### 5.4. Research Limitations and Future Perspectives

This study just determines the assessment of work skill development from the aspect of the students and fails to collect the related data on the teachers. Moreover, considering perception at distinct periods has distinct effects on people's activity and selection, future studies might use a deep interview from the perspective of students or mixed methods. Furthermore, the impact of work skill development on perceived employability is many sided. Future researchers could add dimensions to study variables in areas such as work skills development. The current study just analyses the mediating factors between work skills development and perceived employability. Therefore, future studies should analyze moderators in the research framework.

## Figures and Tables

**Figure 1:** Hypothesis model.

**Figure 2:** The unstandardized path coefficients in model testing. Note: ^*∗∗∗*^*p* < 0.001.

**Table 1:** Model fit.

Model	*χ* ^2^	*df*	*χ* ^2^ */df*	CFI	TLI	AIC	BIC	RMSEA	SRMR
Four-factor model	4098.889	1169	3.506	0.905	0.900	69487.517	70220.831	0.056	0.033
Three-factor model	6944.082	1172	5.925	0.813	0.804	72326.710	73045.922	0.078	0.077
Two-factor model	9742.295	1174	8.298	0.722	0.710	75120.923	75830.734	0.095	0.087
Single-factor model	10586.684	1175	9.010	0.695	0.682	75963.313	76668.422	0.099	0.087

Four-factor model: work skills development, network behavior, decision self-efficacy, and perceived employability. Three-factor model: work skills development + network behavior, decision self-efficacy, and perceived employability. Two-factor model: work skills development + network behavior + decision self-efficacy and perceived employability. Single-factor model: work skills development + networking behaviors + decision self-efficacy + perceived employability.

**Table 2:** Descriptive statistics and correlation.

Variable	Mean	SD	CR	AVE	1	2	3	4
1. Work skills development	3.307	0.645	0.968	0.591	**(0.769)**			
2. Networking behaviors	3.378	0.630	0.931	0.574	0.617^*∗∗*^	**(0.758)**		
3. Decision self-efficacy	3.331	0.583	0.942	0.576	0.641^*∗∗*^	0.666^*∗∗*^	**(0.759)**	
4. Perceived employability	3.275	0.628	0.888	0.532	0.596^*∗∗*^	0.735^*∗∗*^	0.740^*∗∗*^	**(0.729)**

*Note.* ^*∗*^ *p*  <  0.05; ^*∗∗*^*p*  <  0.01. Diagonal number is the square root value of AVE.

**Table 3:** Heterotrait-monotrait ratio statistics (HTMT).

Construct	1	2	3	4
1. Work skills development				
2. Networking behaviors	0.649			
3. Decision self-efficacy	0.671	0.711		
4. Perceived employability	0.643	0.810	0.810	

**Table 4:** Exploratory factor analysis results.

Scales	Items	Factor 1	Factor 2	Factor 3	Factor 4
WSD	WSD1	**0.680**	0.144	0.122	0.230
	WSD2	**0.672**	0.082	0.075	0.251
	WSD3	**0.683**	0.187	0.168	0.135
	WSD4	**0.689**	0.147	0.095	0.223
	WSD5	**0.693**	0.175	0.195	0.202
	WSD6	**0.710**	0.201	0.167	0.150
	WSD7	**0.725**	0.213	0.153	0.135
	WSD8	**0.743**	0.159	0.214	0.183
	WSD9	**0.730**	0.184	0.221	0.194
	WSD10	**0.767**	0.216	0.163	0.142
	WSD11	**0.753**	0.232	0.217	0.111
	WSD12	**0.726**	0.258	0.228	0.110
	WSD13	**0.658**	0.261	0.163	0.030
	WSD14	**0.716**	0.281	0.194	0.057
	WSD15	**0.710**	0.206	0.204	0.094
	WSD16	**0.736**	0.246	0.211	0.026
	WSD17	**0.722**	0.214	0.233	0.129
	WSD18	**0.756**	0.242	0.215	0.085
	WSD19	**0.706**	0.214	0.227	0.130
	WSD20	**0.758**	0.243	0.227	0.080
	WSD21	**0.701**	0.200	0.303	0.122

DSE	DSE1	0.256	**0.575**	0.292	0.384
	DSE2	0.251	**0.612**	0.243	0.358
	DSE3	0.267	**0.629**	0.238	0.345
	DSE4	0.206	**0.675**	0.201	0.197
	DSE5	0.284	**0.725**	0.229	0.170
	DSE6	0.289	**0.711**	0.224	0.142
	DSE7	0.248	**0.697**	0.237	0.141
	DSE8	0.231	**0.732**	0.211	0.092
	DSE9	0.247	**0.600**	0.171	0.264
	DSE10	0.270	**0.705**	0.168	0.120
	DSE11	0.251	**0.695**	0.208	0.166
	DSE12	0.273	**0.685**	0.234	0.129

NB	NB1	0.296	0.220	**0.673**	0.139
	NB2	0.229	0.215	**0.693**	0.145
	NB3	0.314	0.258	**0.653**	0.108
	NB4	0.291	0.254	**0.671**	0.179
	NB5	0.229	0.294	**0.669**	0.132
	NB6	0.210	0.258	**0.716**	0.204
	NB7	0.226	0.209	**0.726**	0.224
	NB8	0.236	0.165	**0.672**	0.289
	NB9	0.218	0.197	**0.659**	0.286
	NB10	0.191	0.214	**0.676**	0.254

PE	PE1	0.188	0.259	0.302	**0.527**
	PE2	0.242	0.227	0.355	**0.558**
	PE3	0.227	0.249	0.309	**0.658**
	PE4	0.255	0.283	0.321	**0.625**
	PE5	0.218	0.377	0.320	**0.614**
	PE6	0.207	0.338	0.310	**0.518**
	PE7	0.216	0.434	0.260	**0.550**

Extraction method: principal component analysis. Rotation method: maximum variance rotation method (Varimax). ^a^The rotation has converged after 6 iterations. *Note.* WSD = work skills development; DSE  =  decision self-efficacy; NB  =  networking behaviors; PE = perceived employability.

**Table 5:** Chain mediating effect.

	Path	Estimation	CI at 95% level	
Total indirect effect		0.502	0.426	0.584
Total effect		0.528	0.453	0.608
Direct effect	WSD⟶PE	0.026	−0.031	0.083
Indirect effect	WSD⟶NB⟶PE	0.241	0.194	0.297
	WSD⟶DSE⟶PE	0.142	0.106	0.184
	WSD⟶NB⟶DSE⟶PE	0.120	0.092	0.156

*Note.* CI, confidence Interval; WSD, work skills development; NB, network behavior; DSE, decision self-efficacy; PE, perceived employability.

## Data Availability

Data from this study are available and support the finding.

## References

[1] Sisodia S., Agrawal N. (2019). Examining employability skills for healthcare services in India: a descriptive literature review. *International Journal of Service Science, Management, Engineering, and Technology*.

[2] Li J., Li J., Jia R., Wang Y., Qian S., Xu Y. (2020). Mental health problems and associated school interpersonal relationships among adolescents in China: a cross-sectional study. *Child and Adolescent Psychiatry and Mental Health*.

[3] Nørgaard B., Ammentorp J., Kyvik K. O., Kofoed P. E. (2012). Communication skills training increases self‐efficacy of health care professionals. *Journal of Continuing Education in the Health Professions*.

[4] Işik E. (2012). The relationship of career decision self-efficacy, trait anxiety, and affectivity among undergraduate students. *Psychological Reports*.

[5] Petruzziello, G., R. Chiesa, and M.G. Mariani (2022). The storm doesn’t touch me!—the role of perceived employability of students and graduates in the pandemic era. *Sustainability*.

[6] Bandaranaike S., Willison J. Work skill development framework: an innovative assessment for work integrated learning.

[7] Fatimah D., Trisnaningsih T., Pujiati P. (2022). Soft skills of SMK IT baitunnur students in dealing with work readiness. *International Journal of Multicultural and Multireligious Understanding*.

[8] Bandaranaike S. The Work Skill Development [WSD] framework: work-ready competencies for today and tomorrow.

[9] Klein E., Lewandowski-Cox J. (2019). Music technology and Future Work Skills 2020: an employability mapping of Australian undergraduate music technology curriculum. *International Journal of Music Education*.

[10] Finch D. J., Hamilton L. K., Baldwin R., Zehner M. (2013). An exploratory study of factors affecting undergraduate employability. *Education + Training*.

[11] Yao C. W., Tuliao M. D. (2019). Soft skill development for employability. *Higher Education, Skills and Work-based Learning*.

[12] Forrier A., Sels L. (2003). The concept employability: a complex mosaic. *International Journal of Human Resources Development and Management*.

[13] Bandura A. (1999). Social cognitive theory: an agentic perspective. *Asian Journal of Social Psychology*.

[14] Berntson E., Marklund S. (2007). The relationship between perceived employability and subsequent health. *Work & Stress*.

[15] Van Dam K. (2004). Antecedents and consequences of employability orientation. *European Journal of Work & Organizational Psychology*.

[16] Bandura A. (2018). Toward a psychology of human agency: pathways and reflections. *Perspectives on Psychological Science*.

[17] Bandura A., Caprara G. V., Barbaranelli C., Gerbino M., Pastorelli C. (2012). Role of affective self regulatory efficacy on diverse spheres of Psychosocial functioning. *Child Development*.

[18] Fugate M., Kinicki A. J., Ashforth B. E. (2004). Employability: a psycho-social construct, its dimensions, and applications. *Journal of Vocational Behavior*.

[19] Gowan M. A., Karren R. (2012). Employability, well‐being and job satisfaction following a job loss. *Journal of Managerial Psychology*.

[20] Hoye G., Hooft E. A. J., Lievens F. (2009). Networking as a job search behaviour: a social network perspective. *Journal of Occupational and Organizational Psychology*.

[21] McDonald S. (2009). Right place, right time: serendipity and informal job matching. *Socio-Economic Review*.

[22] Mouw T. (2003). Social capital and finding a job: do contacts matter?. *American Sociological Review*.

[23] Garg R., Telang R. (2011). To Be or not to Be linked on LinkedIn: job search using online social networks. *SSRN Electronic Journal*.

[24] Bandura A. (1994). Social cognitive theory, some section from Social foundations of thought and action: a social cognitive theory. *Annals of Child Development*.

[25] Granovetter M., Soong R. (2010). Threshold models of diffusion and collective behavior. *Journal of Mathematical Sociology*.

[26] Rogers E. M., Kincaid D. L. (1981). *Communication Networks: Toward a New Paradigm for Research New York, US, Free Press*.

[27] Bandura A. (1991). Social cognitive theory of self-regulation. *Organizational Behavior and Human Decision Processes*.

[28] Locke E. A., Latham G. P. (1990). *A Theory of Goal Setting & Task Performance Hoboken, New Jersey, Prentice-Hall*.

[29] Azjen I. (1981). Attitudes, personality and behavior. *The Journal of Genetic Psychology*.

[30] Rotter J., Feather Em N. T. (1982). Social learning theory. *Expectations and Actions: Expectancy-Value Models in Psychology*.

[31] Vroom V. H. (1964). Work and motivation.

[32] Bandura A. (1997). *Self-efficacy: The Exercise of Control*.

[33] Deigh J. (1985). *Personal being: a Theory for individual psychology*. Rom harré. *Ethics*.

[34] Weiner B. (1986). *An Attributional Theory of Motivation and Emotion*.

[35] Krueger N. F., Dickson P. R. (1993). Perceived self-efficacy and perceptions of opportunity and threat. *Psychological Reports*.

[36] Krueger N., Dickson P. R. (1994). How believing in ourselves increases risk taking: perceived self-efficacy and opportunity recognition. *Decision Sciences*.

[37] Wood R., Bandura A. (1989). Social cognitive theory of organizational management. *Academy of Management Review*.

[38] Debowski S., Wood R. E., Bandura A. (2001). Impact of guided exploration and enactive exploration on self-regulatory mechanisms and information acquisition through electronic search. *Journal of Applied Psychology*.

[39] Sampson R. J., Raudenbush S. W., Earls F. (1997). Neighborhoods and violent crime: a multilevel study of collective efficacy. *Science*.

[40] Chandran A. V. (2019). Employability skills of management students in Bangalore. *SEMCOM Management & Technology Review*.

[41] Rahmat M., Ahmad K., Idris S., Zainal N. F. A. (2012). Relationship between employability and graduates’ skill. *Procedia - Social and Behavioral Sciences*.

[42] Jackson D. (2013). The contribution of work-integrated learning to undergraduate employability skill outcomes. https://files.eric.ed.gov/fulltext/EJ1113705.pdf.

[43] Tamrakar S., Das R. (2016). Effects of local language skills on the employabiblity of International graduates in Norway. https://ntnuopen.ntnu.no/ntnu-xmlui/bitstream/handle/11250/2461878/Tamrakar,%20S.%20og%20Das,%20R.%202016.pdf?sequence=1.

[44] Širca N. T., Nastav B., Lesjak D., Sulčič V. (2006). The labour market, graduate competences and study programme development: a case study. *Higher Education in Europe*.

[45] Wei X., Liu X., Sha J. (2019). How does the entrepreneurship education influence the students’ innovation? Testing on the multiple mediation model. *Frontiers in Psychology*.

[46] Andrews J., Higson H. (2008). Graduate employability, “soft skills” versus “hard” business knowledge: a European study. *Higher Education in Europe*.

[47] Batistic S., Tymon A. (2017). Networking behaviour, graduate employability: a social capital perspective. *Education + Training*.

[48] Chen Y. (2017). Graduate employability: the perspective of social network learning. *Eurasia Journal of Mathematics, Science and Technology Education*.

[49] Craig K. (2021). Perceptions of employability within an undergraduate science department: a case study to define current strategies and recommend improvements. *Journal of Academic Research and Essays*.

[50] Yang L., Aumeboonsuke V. (2022). The impact of entrepreneurial orientation on firm performance: the multiple mediating roles of competitive strategy and knowledge creation process. *Mobile Information Systems*.

[51] Forret M. L., Dougherty T. W. (2004). Networking behaviors and career outcomes: differences for men and women?. *Journal of Organizational Behavior*.

[52] Gibson C., H Hardy III J., Ronald Buckley M. (2014). Understanding the role of networking in organizations. *Career Development International*.

[53] Clements A. J., Kamau C. (2017). Understanding students’ motivation towards proactive career behaviours through goal-setting theory and the job demands–resources model. *Studies in Higher Education*.

[54] Charoensukmongkol P. (2022). Supervisor-subordinate guanxi and emotional exhaustion: the moderating effect of supervisor job autonomy and workload levels in organizations. *Asia Pacific Management Review*.

[55] Makki B. I., Javaid M. U., Bano S. (2016). Level of work readiness skills, career self-efficacy and career exploration of engineering students. *NFC-IEFR Journal of Engineering and Scientific Research*.

[56] Makki B. I., Salleh R., Harun H. Work readiness, career self-efficacy and career exploration: a correlation analysis.

[57] Ahmed H., Nawaz S., Imran Rasheed M. (2019). Self-efficacy, self-esteem, and career success: the role of perceived employability. *Journal of Management Sciences*.

[58] Berntson E., Näswall K., Sverke M. (2008). Investigating the relationship between employability and self-efficacy: a cross-lagged analysis. *European Journal of Work & Organizational Psychology*.

[59] Tentama F., Nur M. Z. (2021). The correlation between self-efficacy and peer interaction towards students’ employability in vocational high school. *International Journal of Evaluation and Research in Education*.

[60] Ngo H.-y., Liu H., Cheung F. (2017). Perceived employability of Hong Kong employees: its antecedents, moderator and outcomes. *Personnel Review*.

[61] Sultana R., Malik O. F. (2020). Protean career attitude, perceived internal employability and perceived external employability; does self-efficacy make a difference. *Middle East J. of Management*.

[62] Charoensukmongkol P., Pandey A. (2020). The influence of cultural intelligence on sales self-efficacy and cross-cultural sales presentations: does it matter for highly challenge-oriented salespeople?. *Management Research Review*.

[63] Brown C., Darden E. E., Shelton M. L., Dipoto M. C. (2016). Career exploration and self-efficacy of high school students: are there urban/suburban differences?. *Journal of Career Assessment*.

[64] Chen S., Chen H., Ling H., Gu X. (2021). How do students become good workers? Investigating the impact of gender and school on the relationship between career decision-making self-efficacy and career exploration. *Sustainability*.

[65] Creed P. A., Patton W., Prideaux L. A. (2007). Predicting change over time in career planning and career exploration for high school students. *Journal of Adolescence*.

[66] Ochs L. A., Roessler R. T. (2016). Predictors of career exploration intentions. *Rehabilitation Counseling Bulletin*.

[67] Kanten S., Kanten P., Yeşiltaş M. (2016). The role of career self-efficacy on the effect of parental career behaviors on career exploration: a study on school of tourism and hotel management’ students. *European Journal of Multidisciplinary Studies*.

[68] Xin L., Tang F., Li M., Zhou W. (2020). From school to work: improving graduates’ career decision-making self-efficacy. *Sustainability*.

[69] Gushue G. V., Whitson M. L. (2016). The relationship among support, ethnic identity, career decision self-efficacy, and outcome expectations in african American high school students. *Journal of Career Development*.

[70] Kezar A., Hypolite L., Kitchen J. A. (2019). Career self-efficacy: a mixed-methods study of an underexplored research area for first-generation, low-income, and underrepresented college students in a comprehensive college transition program. *American Behavioral Scientist*.

[71] Padula M. A. (1994). Reentry women: a literature review with recommendations for counseling and research. *Journal of Counseling and Development*.

[72] Quimby J. L., O’Brien K. M. (2004). Predictors of student and career decision-making self-efficacy among nontraditional college women. *The Career Development Quarterly*.

[73] Zhang Y., Cui L., Zhang G., Sarasvathy S., Anusha R. (2018). An exploratory study of antecedents of entrepreneurial decision-making logics: the role of self-efficacy, optimism, and perspective taking. *Emerging Markets Finance and Trade*.

[74] Pond S. B., Hay M. S. (1989). The impact of task preview information as a function of recipient self-efficacy. *Journal of Vocational Behavior*.

[75] Jimmieson N. L., Terry D. J., Callan V. J. (2004). A longitudinal study of employee adaptation to organizational change: the role of change-related information and change-related self-efficacy. *Journal of Occupational Health Psychology*.

[76] Burt R. S. (1997). A note on social capital and network content. *Social Networks*.

[77] Sparrowe R. T., Liden R. C., Wayne S. J., Kraimer M. L. (2001). Social networks and the performance of individuals and groups. *Academy of Management Journal*.

[78] Marsden P. V. (1988). Homogeneity in confiding relations. *Social Networks*.

[79] Vardaman J. M., Amis J. M., Dyson B. P., Wright P. M., Van de Graaff Randolph R. (2012). Interpreting change as controllable: the role of network centrality and self-efficacy. *Human Relations*.

[80] Yun J., Long W. Thoughts on “going out” of school-enterprise cooperation of higher education in yunnan.

[81] Pop C., Khampirat B. (2019). Self-assessment instrument to measure the competencies of Namibian graduates: testing of validity and reliability. *Studies In Educational Evaluation*.

[82] Lent R. W., Ezeofor I., Morrison M. A., Penn L. T., Ireland G. W. (2016). Applying the social cognitive model of career self-management to career exploration and decision-making. *Journal of Vocational Behavior*.

[83] Rothwell A., Herbert I., Rothwell F. (2008). Self-perceived employability: construction and initial validation of a scale for university students. *Journal of Vocational Behavior*.

[84] Räty H., Hytti U., Kasanen K., Komulainen K., Siivonen P., Kozlinska I. (2019). Perceived employability and ability self among Finnish university students. *European Journal of Psychology of Education*.

[85] Karli U. (2016). Adaptation and validation of self-perceived employability scale: an analysis of sports department students and graduates. *Educational Research and Reviews*.

[86] Vargas R., Sánchez-Queija M. I., Rothwell A., Parra Á. (2019). *Self-perceived Employability in Spain*.

[87] Räty H., Komulainen K., Harvorsén C., Nieminen A., Korhonen M. (2018). University students’ perceptions of their “ability selves” and employability: a pilot study. *Nordic Journal of Studies in Educational Policy*.

[88] Hayes A. F. (2013). *Introduction to Mediation, Moderation, and Conditional Process Analysis: A Regression-Based Approach*.

[89] Hu L. t, Bentler P. M. (1999). Cutoff criteria for fit indexes in covariance structure analysis: conventional criteria versus new alternatives. *Structural Equation Modeling: A Multidisciplinary Journal*.

[90] Zhou H., Long L. (2004). Statistical remedies for common method biases. *Advances in Psychological Science*.

[91] Hair J., Black W., Babin B., Anderson R. (2010). *Multivariate Data Analysis*.

[92] Fornell C., Larcker D. F. (1981). Evaluating structural equation models with unobservable variables and measurement error. *Journal of Marketing Research*.

[93] Henseler J., Ringle C. M., Sarstedt M. (2015). A new criterion for assessing discriminant validity in variance-based structural equation modeling. *Journal of the Academy of Marketing Science*.

[94] St Louis A. T., Thompson P., Sulak T. N., Harvill M. L., Moore M. E. (2021). Infusing 21st century skill development into the undergraduate curriculum: the formation of the iBEARS network. *Journal of Microbiology & Biology Education*.

[95] Crebert G., Bates M., Bell B., Patrick C. J., Cragnolini V. (2004). Developing generic skills at university, during work placement and in employment: graduates’ perceptions. *Higher Education Research and Development*.

[96] Nicholls E., Walsh M., Walsh M. (2007). University of Wolverhampton case study. *Education + Training*.

[97] Gribble C., McRae N. (2017). Creating a climate for global WIL: barriers to participation and strategies for enhancing international students’ involvement in WIL in Canada and Australia. *Professional Learning in the Work Place for International Students*.

